# Ultrasound Elastography supplement assessing nodal status of magnetic resonance imaging staged cervical N0 patients with nasopharyngeal carcinoma

**DOI:** 10.1186/s40644-019-0199-3

**Published:** 2019-03-04

**Authors:** Jian Li, Fei Han, Yunxian Mo, Xindan Chen, Yong Li, Feifei Zuo

**Affiliations:** 1 Department of Diagnostic and Interventional Ultrasound, Sun Yat-Sen University Cancer Center, State Key Laboratory of Oncology in South China, Collaborative Innovation Center for Cancer Medicine, No.651, Dong-feng-dong Road, Guangzhou, 510060 China; 2 Department of Radiation Oncology, Sun Yat-Sen University Cancer Center, State Key Laboratory of Oncology in South China, Collaborative Innovation Center for Cancer Medicine, No.651, Dong-feng-dong Road, Guangzhou, 510060 China; 3 Department of Radiology, Sun Yat-Sen University Cancer Center, State Key Laboratory of Oncology in South China, Collaborative Innovation Center for Cancer Medicine, No.651, Dong-feng-dong Road, Guangzhou, 510060 China; 4 Department of Pathology, Sun Yat-Sen University Cancer Center, State Key Laboratory of Oncology in South China, Collaborative Innovation Center for Cancer Medicine, No.651, Dong-feng-dong Road, Guangzhou, 510060 China

**Keywords:** Ultrasound, Shear wave Elastography, Nasopharyngeal carcinoma, Small lymph node, Diagnostic performance

## Abstract

**Background:**

To determine whether ultrasound elastography can distinguish reactive or metastatic small lymph nodes (sLN) of magnetic resonance imaging (MRI) staged cervical N0 patients with nasopharyngeal carcinoma (NPC).

**Methods:**

A pilot study was performed involving the diagnostic performances of conventional high-frequency ultrasound (CHFU) and/or shear wave elastography (SWE) for predicting metastases in sLN of MRI-staged N0 NPC patients with reference to the histologically-proven ultrasound guided core needle biopsy (US-CNB). The diagnosis of CHFU was based on the superficial lymph node ultrasonic criteria with the five-point-scale (FPS). The mean (Emean), minimum (Emin) and maximum (Emax) of the elasticity indices were measured by SWE at the stiffest part of the sLN in kilopascal. Diagnostic performances were analyzed using a receiver operating curve (ROC) on a per-node basis. The authenticity of this article has been validated by uploading the key raw data onto the Research Data Deposit public platform (http://www.researchdata.org.cn), with the approval RDD number as RDDA2017000447.

**Results:**

All 113 cervical sLN of 49 MRI-staged cervical N0 NPC patients underwent evaluation of CHFU and SWE; 38 sLN (FPS < 2) were regarded as benign, which were excluded from subsequent analysis due to none biopsy-proven. And 75 indeterminate sLN (FPS ≥ 2) were referred to US-CNB and revealed 15 (20%) metastases. All SWE elastic indices were significantly higher in malignant sLNs than in benign sLNs (*p* < 0.05). Moreover, Emax exhibited the highest diagnostic value (AUC:0.733 ± 0.067, *p* = 0.005) with excellent measurement reproducibility (ICC: 0.786; 95%CI: 0.684, 0.864). CHFU plus SWE was superior to CHFU or SWE alone for predicting metastases in sLN of MRI-staged N0 patients with NPC (*p* < 0.001).

**Conclusions:**

CHFU plus SWE is an optional non-invasive modality to supplement MRI in assessing cervical nodal status of patients with NPC.

**Electronic supplementary material:**

The online version of this article (10.1186/s40644-019-0199-3) contains supplementary material, which is available to authorized users.

## Background

Nasopharyngeal carcinoma (NPC), an endemic disease in Southeast Asia, is a non-lymphomatous squamous-cell carcinoma that occurs in the epithelial lining of the nasopharynx with a distinct epidemiology, etiology and clinical manifestation compared with other head and neck cancers. [1, 2] NPC has the highest prevalence of regional lymph nodes metastasis among head and neck cancers, often bilaterally spreads to retropharyngeal, upper jugular, and spinal accessory nodes. [3] Radiation is the primary treatment for nasopharyngeal lesion and cervical lymph nodes metastasis based on magnetic resonance imaging (MRI) staging. [4] Even for NPC patients with clinically negative neck lymph nodes, elective and prophylactic irradiations to whole neck or upper neck are necessary; this implies that occult metastasis may exist in regional nodes of patients that are clinically staged as N0. [5] Ultrasound-guided core needle biopsy (US-CNB) of indeterminate lymph nodes is a standard practice to harvest sufficient tissue for histologically verifying cervical lymph nodes metastases of patients with NPC due to being convenient, real-time imaging guidance and being minimally invasive. [6]

Non-invasive characterization of cervical small lymph nodes (sLN) is challenging. The determination of malignant cervical lymph nodes primarily depends on the radiological criteria of the minimum axis ≥ 10 mm in the transverse plane, as well as on evidence of central necrosis or extra-capsular spread in MRI or CT. [7] MRI is the primary approach to diagnose node metastasis and is superior to CT for staging NPC. [8] Diffusion-weighted MRI is feasible for differentiating metastatic from non-metastatic nodes in NPC patients with high accuracy. [9] A previous study found that positron emission tomography/computed tomography detects more distant metastases than conventional staging in patients with NPC, while it is limited in detecting metastatic sLN. [10, 11] Conventional high-frequency ultrasonography (CHFU) with B mode and color Doppler flow imaging were used for evaluation of cervical lymph nodes for several decades. In addition, the ultrasound features including Doppler findings of malignancy in macro-metastatic lymph nodes are well-known. [12] However, it is more difficult to determine whether malignancy is present in sLN. Contrast-enhanced ultrasound, which allows for visualization of lymph node micro-vessels, demonstrated centripetal inhomogeneous enhancement with perfusion defects in malignant lymph nodes that was distinct from the centrifugal homogeneous enhancement of benign lymph nodes, although the results were inconsistent. Moreover, the injection of contrast media is needed, and the radiologist should be experienced in contrast-enhanced ultrasound. [13, 14] Elastography-based imaging techniques have received substantial attention in recent years for non-invasive assessment of tissue mechanical properties. [15] Ultrasound Elastography is divided into string elastography and shear wave elastography (SWE). [16] Metastatic lymph nodes appear to be much stiffer compared with the adjacent soft tissue or benign lymph nodes. Compared with strain elastography using hand compression, SWE based on supersonic shear imaging can quantitatively measure the velocity in real-time and indirectly measure the stiffness in KiloPascals (kPa) with more reproducibility. [17, 18] The most recent meta-analysis showed that SWE is an acceptable modality for diagnosing malignant cervical lymph nodes, and demonstrated a summary sensitivity of 81% and specificity of 85%. [19] And, SWE is a reproducible quantitative tool that can be used to characterize sLN of patients with NPC. [18]

The prevalence of metastasis in cervical sLN of MRI-staged cervical N0 patients with NPC is unclear, and the detection of metastasis in these sLN could benefit precision radiotherapy. The purpose of the present study is to evaluate the effectiveness of CHFU plus SWE as a diagnostic tool to supplement MRI in assessing cervical nodal status, and to elucidate the prevalence of metastasis in cervical sLN in MRI-staged cervical N0 patients with NPC.

## Material and methods

### Study population

This prospective study was performed at Sun Yat-Sen University Cancer Center with approval (YB2014–26) from the Institutional Review Board Ethical and Research Committee during May 2014 to April 2016. Written informed consent was obtained from all enrolled patients.

Eligibility criteria were as follows: initially diagnosed patients with NPC confirmed by nasopharyngeal scope guided biopsy; MRI imaging of head and neck in a week of the initial diagnosis showed no metastatic cervical lymph nodes based on the radiologic size criteria using 1 .5T MRI system (MAGNETOM Aera, Siemens Healthineers); [20] was defined as MRI-staged cervical N0 with independence of the retropharyngeal node status; no distant metastasis; no previous cervical radiation or surgery; no history of another malignant tumor; having the ability to undergo subsequent radiation-centered therapy. Exclusion criteria included US-CNB failure with no metastatic or lymphatic tissue found in the biopsy sample, or lost to imaging follow-up in two years.

### Ultrasound Elastography protocol

CHFU and SWE were performed in all patients by radiologists with more than 10 years of experience in ultrasonic diagnosis, using only Real-time ShearWave™ Elastography device (Aixplorer®, Supersonic Imagine, Provence, France) with a conventional 15–4 MHz transducer linear probe (SuperLinear™ SL15–4) within 3 days of head and neck MRI. sLN were defined according to the sizes of their minimum axial diameter (> 3 mm; ≤10 mm) in the maximum longitudinal US section. Regional distribution was determined according to the consensus guidelines of the lymph node levels. [21] The evaluation of cervical sLN by CHFU and SWE was done as described by Desmots F. et al. [22] During measurement of SWE, an appropriate region of interest (ROI; long: 20 mm; wide: 20 mm) covered the entire target sLN and a small amount of surrounding tissue. The measurements were taken 3 times to assess the reproducibility. Three Q-boxes (trademark by Supersonic, Imagine, Inc.) 3 mm in diameter were placed on the visibly stiffest region in the node. The device automatically generated several elasticity indices for each Q-box: mean (Emean), minimum (Emin) and maximum (Emax) elasticity values in kPa, as shown in Fig. 1 and Fig. 2.

**Fig. 1:** A benign cervical sLN of a 40-year-old woman with nasopharyngeal carcinoma. **a** Axial T2-weighted MRI reveals an 8.0 × 11.0-mm-sized lymph node in the left level II a (green arrow). **b** Conventional high-frequency ultrasonography with B mode imaging demonstrating shift of hyper-echoic hilum, inhomogeneous internal echogenicity and regular margins. **c** Normal hilar vascularization is not seen in color Doppler. **d** Shear wave elastography (above) is displayed along with B-mode image (down) simultaneously on the same screen. The node displays relatively homogeneous blue color elasticity signal. **e** Ultrasound guided core needle biopsy of the targeted sLN. White triangles represent the needle. Green arrow represents the targeted sLN. **f** Hematoxylin and eosin staining (magnification 100×) of the core needle biopsy showed normal lymphatic tissue and no malignancy. sLN denoted small lymph node

**Fig. 2:** A metastatic cervical small lymph node of a 30-year-old man with nasopharyngeal carcinoma. **a** Axial T2-weighted MR image reveals an 8.0 × 10.0-mm-sized lymph node in the left level IIb area (green arrow). **b** Appearance in Conventional high-frequency ultrasonography B mode with displacement of hilum, heterogeneous internal echogenicity and irregular margins. **c** Abnormal peripheral vascularization is seen in color Doppler. **d** Shear wave elastography reveals markedly heterogeneous color equating to very high and low stiffness in the node. Shear elasticity indices of the stiffest region were measured by one 3-mm diameter Q-box. **e** Ultrasound guided core needle biopsy of the targeted stiffest area of sLN revealed by shear wave elastography. White triangles showed the needle. Green arrow showed the targeted small lymph node. **f** Hematoxylin and eosin staining (magnification 100×) of the core needle biopsy sample showed that metastasis from nasopharyngeal carcinoma in the lymph node, which was confirmed by immune-histo-chemistry

### US-CNB and histopathology evaluation

The sLN were graded on the five-point-scale (FPS), in accordance to the criteria of conventional ultrasound diagnosis for superficial lymph nodes. [12] Points were determined by five criteria: minor axis (diameter ≥ 6.5 mm, 1 point; diameter < 6.5 mm, 0 point); the ratio of Long axis/Short axis (L/S) (ratio ≤ 2, 1 point; ratio > 2, 0 point); the border (irregular, 1 point; regular, 0 point); echogenicity of cortex (inhomogeneous, 1 point; homogeneous, 0 point); and hilum (disappearance or displacement, 1 point, present in the center, 0 point). The corresponding grades for the total points were as follows: 1 = lack of malignancy, point 0; 2 = in favor of the absence of malignancy, point 1; 3 = doubtful malignancy, point 2; 4 = highly probable malignancy, point 3; 5 = obvious signs of malignancy, point 4 or 5. FPS < 2 was determined as benign lymph nodes with imaging follow-up and those nodes were excluded from subsequent analysis, while FPS ≥ 2 was determined as indeterminate lymph nodes with US-CNB.

An ultrasonography system (Avius, Hitachi, Tokyo, Japan) with a 13.0 MHz transducer (EUP-L74 M, Hitachi, Tokyo, Japan) was used for the biopsy. The information obtained from MRI, CHFU and SWE was used to optimize and plan the biopsy route and target. The Q-box exhibiting the highest value was regarded as the target area. A 16-gauge core biopsy needle (Magnum; Bard, Covington, GA, USA) was used for the US-CNB after routine sterilization and local anesthesia (3–5 ml 1% Lidocaine). A free hand approach was used for the CNB procedure with real-time US monitoring. 2–3 core biopsies of the lymph nodes were performed. The specimens were fixed in 10% formalin and were sent to the pathology department for evaluation. The patients stayed in the observation room for at least 15 min due to possible morbidities.

Core needle biopsy specimens were stained with routine hematoxylin and eosin (H & E). All results that described staining patterns or morphologic features of the specimens were evaluated under the guidance of an experienced pathologist specialized in cancer pathology. Metastases from NPC or lymphatic tissue in the sample of US-CNB were adequate pathology reports.

### Treatment and follow-up

All enrolled patients underwent radiation-centered therapy. The cervical lymph nodes status was evaluated by MRI and CHFU every 6 months post-radiotherapy in the first two years and then annually thereafter.

### Statistics

All statistical analyses were performed using SPSS (version 23.0, IBM, Armonk, New York). The measurement reproducibility was estimated with two-way mixed intra-class correlation coefficient (ICC) test in reliability analysis, Value greater than 0.75 indicated excellent agreement. To evaluate the correlation between ultrasonic findings, SWE and the pathologic findings of a particular lymph node were performed on a per-node basis. Comparisons of quantitative data between benign and metastatic pathologies were performed using the Mann-Whitney U test. Receiver operator characteristic (ROC) curves were constructed using biopsy pathological diagnosis as the reference standard. The area under the curve (AUC) was then calculated. For quantitative variables, the Youden method was used to determine the optimal cut-off values in association with nodes status, and the corresponding sensitivity, specificity, accuracy, positive predictive values and negative predictive values were generated. McNemar test was used to compare the diagnostic performances of CHFU, SWE, and CHFU plus SWE. For all tests, *p* values < 0.05 were considered statistically significant.

## Results

### General

Fifty-one eligible MRI-staged cervical N0 patients were registered; 2 patients were excluded due to unadequacy of core needle biopsy; 49 patients were enrolled in the present study, of whom 36 were men and 13 were women, with a mean age of 45.2 years old (range, 31.0–58.0 years); 25 patients (25/49, 51.0%) were diagnosed with retro-pharyngeal lymph node metastasis by MRI. A total of 113 sLN were evaluated by CHFU and SWE; 57 sLN were located on the left (9 in Level I; 45 in Level II; 2 in Level III; 1 in Level V), while 56 sLN located on the right (9 in Level I; 41 in Level II; 4 in Level III; 1 in level IV; 1 in Level V); 86 (86/113, 76.1%) sLN were localized in cervical level II. All patients had at least one sLN with FPS ≥ 2.

All 113 sLN were divided into benign sLN (FPS < 2, *n* = 38) and indeterminate sLN (FPS ≥ 2, *n* = 75). The indeterminate sLN (FPS ≥ 2, n = 75) underwent US-CNB for histological diagnosis and showed metastatic sLN (*n* = 15) in 12 patients (12/49, 24.5%); 13 metastatic (13/15, 86.7%) sLN were localized in cervical level II; With the supplement of SWE and US-CNB, 9 patients found 1 metastatic node, of them, 4 patients were upstaged from N0 to N1, 5 patients with retro-pharyngeal lymph node metastasis stayed as N1.Three patients found 1 metastatic node in both sides and were upstaged from N1 to N2; All patients were followed up from 24 months to 47 months (mean, 38; standard deviation, 14) after radiation-centered therapy. No recurrence, cervical sLN progression or distant metastases were observed in the follow-up. The study flow chart is shown in Fig. 3.

**Fig. 3:** Flow chart of this pilot study. CHFU denoted conventional high-frequency ultrasound; SWE denoted shear wave elastography; sLN denoted small lymph nodes; US-CNB denoted ultrasound guided core needle biopsy; MRI denoted magnetic resonance imaging; n denoted number of lymph nodes; N denoted number of patients

### SWE measurement reproducibility

>The ICC of the three measurements of Emax, Emean and Emin was 0.786 (95%CI: 0.684, 0.864), 0.745 (95% CI: 0.628, 0.836) and 0.762 (95%CI: 0.652, 0.848), respectively.

### Morphological features of CHFU, SWE elastic indices and metastatic status of the cervical sLN

The long axis of the benign and metastatic nodes ranged from 5 mm to 32 mm and 10 mm to 20 mm, respectively. The minor axis of the benign and metastatic nodes ranged from 3 mm to 10 mm and 5 mm to 10 mm, respectively. Sixty-two (62/75, 82.7%) sLN did not demonstrate any blood signals, and residence index was not analyzed. Calcification and cystic content were not found in all sLN. Significant differences were observed in the hilum, cortex, ratio of long axis/minor axis, shape, minor axis, and grade based on FPS between metastatic and non-metastatic sLN; The Emax, Emin and Emean were significantly higher in malignant sLN than in benign sLN; which were shown in Table 1. The cut-values of Emax, Emin and Emean for diagnosis of metastatic lymph nodes were 23.33, 7.60 and 16.07, respectively, as calculated by the Youdon method, as shown in Table 2.

**Table 1:** The CHFU morphologic features, SWE elastic indices and metastatic status of 75 indeterminate cervical sLN in 49 patients with nasopharyngeal carcinoma

Characteristics		Metastatic status		*p* value
		Positive *n* = 15	Negative *n* = 60	
shape	oval	3	2	0.021
	Round -like	12	58	
boundary	sharp	10	46	0.426
	indistinct	5	14	
Long axis (mm)	mean ± SD	13.87 ± 2.88	14.4 ± 5.12	0.682
	≥10.5	14	45	0.868
	<10.5	1	15	
Minor axis (mm)	mean ± SD	7.67 ± 1.92	6.30 ± 2.01	0.021
	≥6.5	11	25	0.023
	<6.5	4	35	
Long axis/minor axis	≤2	13	23	0.008
	>2	2	37	
Hilum	Normal	2	42	< 0.001
	Shift or disappear	13	18	
Inhomogeneous thickening of the cortex	Yes	14	31	0.003
	No	1	29	
Blood flow signals	with	0	13	0.047
	without	15	47	
Five-point-scale	=2	1	31	0.002
	> 2	14	29	
Emax (kPa)	mean ± SD	42.34 ± 26.21	22.85 ± 9.95	< 0.001
Emin (kPa)	mean ± SD	14.12 ± 8.96	8.75 ± 4.53	0.002
Emean (kPa)	mean ± SD	32.69 ± 21.03	12.93 ± 6.13	< 0.001

CHFU = conventional high-frequency ultrasound; sLN = small lymph node; SD = standard deviation

**Table 2:** Elastic indices of shear wave elastography and metastatic status of 75 small cervical lymph nodes in 49 nasopharyngeal carcinoma patients who were histologically verified by ultrasound-guided core needle biopsy

Categories of SWE	mean ± SD (kPa)	Cut-value (kPa)	N of ≥Cut-value (positive/negative)	N of <Cut-value (positive/negative)	*p* value
Emax	26.75 ± 16.45	23.33	13/24	2/36	0.001
Emin	9.82 ± 6.02	7.60	13/30	2/30	0.018
Emean	17.82 ± 10.14	16.07	12/20	3/40	0.001

SWE: shear wave elastography; SD: standard deviation; Emax: the maximum of elasticity indices; Emean: the mean of elasticity indices; Emin: the minimum of elasticity indices

### The diagnostic performance of morphological features of CHFU and elastic indices for cervical sLN metastasis

For predicting cervical sLN metastasis, the diagnostic performance of the characteristic of hilum was superior to that of other ultrasonic characteristics or grade of FPS based on CHFU, as shown in Table 3. And the diagnostic performances of Five-Point-Scale scores for characterizing cervical sLN at different cut-off point showed the optimal cut-off point was at 3 (=2 vs > 2). An additional file shows this in more detail [see Additional file 1]. The diagnostic performance of Emax had no significant differences with that of Emean(*p* = 0.709). Both Emax and Emean were superior to Emin (*p* < 0.05). The diagnostic performances of Emax, Emin and Emean were showed in Table 3.

**Table 3:** the diagnostic performances of the characteristics of conventional high-frequency ultrasound and elastic indices of shear wave elastography for metastatic small cervical lymph nodes in nasopharyngeal carcinoma patients

Characteristics	Area Under Curve (mean ± SD)	Sensitivity (%)	Specificity (%)	Positive Predictive Value (%)	Negative Predictive Value (%)	Accuracy (%)	*p* Value	95% C.I. Lower-Upper
Shape	0.583 ± 0.089	20.0	97.7	60.0	83.3	81.3	0.321	0.409–0.758
Boundary	0.550 ± 0.086	33.3	77.7	26.3	82.1	68.0	0.551	0.382–0.718
Long axis (mm)	0.592 ± 0.077	93.3	25.0	24.7	94.8	39.7	0.275	0.443–0.740
Minor axis (mm)	0.658 ± 0.071	73.3	58.3	31.6	90.7	61.3	0.059	0.507–0.809
Long axis/minor axis	0.692 ± 0.073	87.0	58.3	36.4	95.1	67.7	0.022	0.549–0.835
Hilum	0.783 ± 0.063	87.7	70.0	42.9	95.5	73.3	0.001	0.660–0.907
Inhomogeneous thickening of the cortex	0.708 ± 0.065	93.3	48.3	31.1	97.7	57.3	0.013	0.581–0.386
Blood flow signals	0.608 ± 0.073	100.0	22.7	24.2	100.0	37.3	0.197	0.466–0.751
Five-point-scale (=2 vs > 2)	0.725 ± 0.064	93.3	52.7	33.6	97.9	60.0	0.007	0.600–0.850
Emax (kPa)	0.733 ± 0.067	87.7	60.0	35.1	95.7	65.3	0.005	0.602–0.824
Emin (kPa)	0.683 ± 0.071	86.7	50.0	30.2	93.8	57.3	0.018	0.545–0.822
Emean (kPa)	0.784 ± 0.067	80.0	66.7	37.5	93.0	69.3	0.001	0.595–0.872

### The diagnostic performance of CHFU (FPS > 2), SWE (Emax), and CHFU (FPS > 2) plus SWE (Emax) for predicting metastatic cervical sLN

The diagnostic performance of CHFU (FPS > 2) had no significant difference with that of Emax (*p* = 0.405). CHFU (FPS > 2) combined with SWE (Emax) is superior to CHFU (FPS > 2) or SWE (Emax) alone for predicting metastases in cervical sLN (*p* < 0.001), as shown in Fig. 4.

**Fig. 4:** The receiver operating curves and diagnostic performances of CHFU-FPS (> 2), Emax, and CHFU-FPS (> 2) plus Emax in predicting metastasis in 75 cervical small lymph nodes of 49 MRI-staged cervical N0 patients with nasopharyngeal carcinoma

## Discussion

This prospective study, unlike previous studies which had a significant selection bias due to a high proportion of malignant cases (> 50%) [16], initially revealed approximately 24.5% metastases in MRI-staged cervical N0 patients with NPC, and this preliminary result should be reported promptly. The discrepancy with the high prevalence (80%) of node metastases in initial NPC can be due to the study population being mostly focused on the MRI-staged cervical N0 patients. Most metastatic sLN were located in Level II, which was shown in a previous study. [3]

We confirmed that the morphologic features of CHFU, including the shift or disappearance of hilum, short axis, long axis/short axis, and inhomogeneous thickening of cortex, are of value in diagnosis of sLN metastases. Although the diagnostic performance of the single characteristic of the hilum is superior to that of other ultrasonic characteristics or FPS based on the morphologic criteria of CHFU, it is difficult to ensure its consistency with other studies since it is non-quantitative. [12] Only the grade of FPS (> 2) based on ultrasonic characteristics is considered in predicting sLN metastases. The values of SWE modulus were significantly higher in malignant sLN than in benign sLN. Emax was regarded as an optional elastic index with excellent agreement in measurement reproducibility, and was logistically selected as the representative elastic index for characterizing sLN in the current study. No imaging study as of yet identified the occult metastasis or microscopic foci in regional nodes. And we found that CHFU plus SWE is useful to distinguish reactive and malignant sLN.

In the current study, the restaged N0–1 patients underwent upper neck radiation; the upstaged N2 patients underwent whole neck radiation. The upstaged patients received more precise radiation therapy with concurrent chemotherapy, and the follow-up revealed no disease progression. This implied that additional evaluation of CHFU plus SWE can supplement MRI staging of patients with NPC, while benefitting the radiation strategy and prognosis with precise re-staging.

Although micrometastasis can be missed by sampling errors, for patients with NPC whose pre-radiation staging depends on radiology and not surgery, US-CNB can be superior to FNA for diagnosing the metastatic status of cervical sLN due to sufficient tissue and a low false-negative rate. [23]. A notable limitation is that the exact elastography number varies in different manufacturers, and kPa (not m/s) was selected for present study, so this number cannot be applied universally. We selected and recorded one Q-box with a diameter of 3 mm that exhibited the highest value for subsequent analyses instead of averaging all Q-box readings or evaluating the whole node with a single large Q-box; this was because the nodes may exhibit focal spatial heterogeneity due to incomplete infiltration by tumor cells. [24] The Q-box with 3 mm diameter that exhibited the highest value was regarded as the target area in the subsequent US-CNB. And a relatively large number of cervical sLN (*n* = 75) were assessed with SWE to demonstrate the usefulness of targeting the appropriate area of LN for biopsy and influencing the management.

Overall, SWE significantly increases the specificity rate and improves the selection of metastatic node compared to morphologic changes of CHFU alone; therefore, it improves the confidence of the final diagnosis of sLN metastasis; SWE may also be able to select eligible nodes and even the targeted area of the node for biopsy.

## Conclusions

Ultrasound elastography is an optional non-invasive imaging modality that supplements MRI in assessing cervical nodal status in patients with NPC.

## Additional file

Additional file 1: Diagnostic performances of Five-Point-Scale scores for characterizing cervical small lymph node metastasis at different cut-off point. The diagnostic performances of Five-Point-Scale scores for characterizing cervical sLN at different cut-off point showed the optimal cut-off point was at 3 (=2 vs > 2). (DOCX 15 kb)

## Abbreviations

CHFU: conventional high-frequency ultrasound
CT: computerized tomography
Emax: The maximum of the elasticity indices
Emean: The mean of the elasticity indices
Emin: The minimum of the elasticity indices
FPS: Five-point scale
MRI: Magnetic resonance imaging
NPC: Nasopharyngeal carcinoma
ROC: Receiver operating curve
sLN: Small lymph node
SWE: Shear wave elastography
US-CNB: Ultrasound-guided core needle biopsy

## References

[1] Chang ET, Adami HO (2006). The enigmatic epidemiology of nasopharyngeal carcinoma. Cancer epidemiology, biomarkers & prevention : a publication of the American Association for Cancer Research, cosponsored by the American Society of Preventive. Oncology.

[2] Wei WI, Sham JS (2005). Nasopharyngeal carcinoma. Lancet.

[3] Wang X, Hu C, Ying H, He X, Zhu G, Kong L (2015). Patterns of lymph node metastasis from nasopharyngeal carcinoma based on the 2013 updated consensus guidelines for neck node levels. Radiotherapy and oncology : journal of the European Society for Therapeutic Radiology and Oncology.

[4] Chen L, Liu LZ, Chen M, Li WF, Yin WJ, Lin AH (2012). Prognostic value of subclassification using MRI in the t4 classification nasopharyngeal carcinoma intensity-modulated radiotherapy treatment. Int J Radiat Oncol Biol Phys.

[5] Zeng L, Sun XM, Chen CY, Han F, Huang Y, Xiao WW (2014). Comparative study on prophylactic irradiation to the whole neck and to the upper neck for patients with neck lymph node-negative nasopharyngeal carcinoma. Head & neck.

[6] Kim BM, Kim EK, Kim MJ, Yang WI, Park CS, Park SI (2007). Sonographically guided core needle biopsy of cervical lymphadenopathy in patients without known malignancy. Journal of ultrasound in medicine : official journal of the American Institute of Ultrasound in Medicine.

[7] Ng WT, Lee AW, Kan WK, Chan J, Pang ES, Yau TK (2007). N-staging by magnetic resonance imaging for patients with nasopharyngeal carcinoma: pattern of nodal involvement by radiological levels. Radiotherapy and oncology : journal of the European Society for Therapeutic Radiology and Oncology.

[8] Liao XB, Mao YP, Liu LZ, Tang LL, Sun Y, Wang Y (2008). How does magnetic resonance imaging influence staging according to AJCC staging system for nasopharyngeal carcinoma compared with computed tomography?. Int J Radiat Oncol Biol Phys.

[9] Li H, Liu XW, Geng ZJ, Wang DL, Xie CM (2015). Diffusion-weighted imaging to differentiate metastatic from non-metastatic retropharyngeal lymph nodes in nasopharyngeal carcinoma. Dento maxillo facial radiology.

[10] Tang LQ, Chen QY, Fan W, Liu H, Zhang L, Guo L (2013). Prospective study of tailoring whole-body dual-modality [18F]fluorodeoxyglucose positron emission tomography/computed tomography with plasma Epstein-Barr virus DNA for detecting distant metastasis in endemic nasopharyngeal carcinoma at initial staging. Journal of clinical oncology : official journal of the American Society of Clinical Oncology.

[11] Ng SH, Chan SC, Yen TC, Chang JT, Liao CT, Ko SF (2009). Staging of untreated nasopharyngeal carcinoma with PET/CT: comparison with conventional imaging work-up. Eur J Nucl Med Mol Imaging.

[12] Ying M, Bhatia KS, Lee YP, Yuen HY, Ahuja AT (2014). Review of ultrasonography of malignant neck nodes: greyscale, Doppler. contrast enhancement and elastography Cancer imaging : the official publication of the International Cancer Imaging Society.

[13] de Stefano G, Scognamiglio U, Di Martino F, Parrella R, Scarano F, Signoriello G (2016). The role of CEUS in characterization of superficial lymph nodes: a single center prospective study. Oncotarget.

[14] Sato T, Takemura T, Ouchi T, Mori S, Sakamoto M, Arai Y (2017). Monitoring of blood vessel density using contrast-enhanced high frequency ultrasound may facilitate early diagnosis of lymph node metastasis. J Cancer.

[15] Ophir J, Cespedes I, Ponnekanti H, Yazdi Y, Li X (1991). Elastography: a quantitative method for imaging the elasticity of biological tissues. Ultrason Imaging.

[16] Sigrist RMS, Liau J, Kaffas AE, Chammas MC, Willmann JK (2017). Ultrasound Elastography: review of techniques and clinical applications. Theranostics.

[17] Mun HS, Choi SH, Kook SH, Choi Y, Jeong WK, Kim Y (2013). Validation of intra- and interobserver reproducibility of shearwave elastography: phantom study. Ultrasonics.

[18] Chen BB, Li J, Guan Y, Xiao WW, Zhao C, Lu TX (2018). The value of shear wave elastography in predicting for undiagnosed small cervical lymph node metastasis in nasopharyngeal carcinoma: a preliminary study. Eur J Radiol.

[19] Suh CH, Choi YJ, Baek JH, Lee JH (2017). The diagnostic performance of shear wave elastography for malignant cervical lymph nodes: a systematic review and meta-analysis. Eur Radiol.

[20] Tao CJ, Liu X, Tang LL, Mao YP, Chen L, Li WF (2013). Prognostic scoring system for locoregional control among the patients with nasopharyngeal carcinoma treated by intensity-modulated radiotherapy. Chinese journal of cancer.

[21] Gregoire V, Ang K, Budach W, Grau C, Hamoir M, Langendijk JA (2014). Delineation of the neck node levels for head and neck tumors: a 2013 update. DAHANCA, EORTC, HKNPCSG, NCIC CTG, NCRI, RTOG, TROG consensus guidelines. Radiotherapy and oncology : journal of the European Society for Therapeutic Radiology and Oncology.

[22] Desmots F, Fakhry N, Mancini J, Reyre A, Vidal V, Jacquier A (2016). Shear wave Elastography in head and neck lymph node assessment: image quality and diagnostic impact compared with B-mode and Doppler ultrasonography. Ultrasound Med Biol.

[23] Chan JY, Chan RC, Chow VL, To VS, Wei WI (2013). Efficacy of fine-needle aspiration in diagnosing cervical nodal metastasis from nasopharyngeal carcinoma after radiotherapy. Laryngoscope.

[24] Bhatia KS, Cho CC, Tong CS, Yuen EH, Ahuja AT (2012). Shear wave elasticity imaging of cervical lymph nodes. Ultrasound Med Biol.

